This article has been retracted.

# Effect of Evodiamine on Collagen-Induced Platelet Activation and Thrombosis

**DOI:** 10.1155/2022/4893859

**Published:** 2022-07-27

**Authors:** Xiaona Yang, Min Leng, Lihong Yang, Yunzhu Peng, Jing Wang, Qian Wang, Kun Wu, Junhua Zou, Wen Wan, Longjun Li, Yujia Ye, Zhaohui Meng

**Affiliations:** Laboratory of Molecular Cardiology, Department of Cardiology, The First Affiliated Hospital of Kunming Medical University, Kunming, China

## Abstract

Evodia rutaecarpa has multiple pharmacological effects and is widely used in the prevention and treatment of migraine, diabetes, cardiovascular disease, cancer, and other chronic diseases; however, the pharmacological effects of its active compound evodiamine (Evo) have not been thoroughly investigated. The purpose of this study was to investigate the effects of Evo on antiplatelet activation and thrombosis. We discovered that Evo effectively inhibited collagen-induced platelet activation but had no effect on platelet aggregation caused by activators such as thrombin, ADP, and U46619. Second, we found that Evo effectively inhibited the release of platelet granules induced by collagen. Finally, evodiamine inhibits the transduction of the SFKs/Syk/Akt/PLC*γ*2 activation pathway in platelets. According to in vivo studies, Evo significantly prolonged the mesenteric thromboembolism induced by ferric chloride and had no discernible effect on the coagulation function of mice. In conclusion, the antiplatelet and thrombotic effects of Evo discovered in this study provide an experimental basis for the investigation of the pharmacological mechanisms of Evo and the development of antiplatelet drugs.

## 1. Introduction

Ischemic cardiomyopathy and ischemic stroke are the leading causes of death and disability in the world after cancer, accounting for approximately 17 million deaths annually [1–3]. Arterial thrombosis is the primary pathophysiological cause of ischemic cardiomyopathy and ischemic stroke. The primary pathological changes that lead to acute thrombosis are atherosclerotic plaque rupture or vascular endothelial cell injury. Platelets are small fragments of cytoplasm derived from mature megakaryocytes (without nuclei) in the bone marrow. In the resting state, platelets appear as double concave discs and do not interact with the intact vascular wall [4]. Blood clots are damaged during the circulation of blood and eventually form blood clots with blood matrix proteins [5]. Antiplatelet therapy is a crucial intervention for the clinical treatment and prevention of thrombosis [4].

After vascular wall injury, collagen and the von Willebrand factor (VWF) interact with platelets, and platelet membrane complex glycoprotein (GP)Ib-V-IX mediates platelet acute adhesion to the injured surface of the vascular wall under high shear stress [6, 7]. Platelet membrane protein GPVI, integrin *α*2*β*1, and integrin *α*5*β* are expressed following adhesion. The stable adhesion of platelets is mediated by the interaction between 1 and fibrinogen [7]. Platelets adhering to the damaged surface activate platelets further by releasing soluble activators such as ADP and thromboxane, which interact with platelet surface receptors such as thromboxane, purinoreceptors 1 and 12 (P2Y1 and P2Y12), and PAR1 or PAR4 [8–10]. Eventually, the conformation of GPIIb/IIIa, the primary platelet adhesion receptor, changes. GPIIb/IIIa binds to fibronectin with varying degrees of affinity, ultimately promoting stable platelet aggregation and thrombosis [11].

Evodia rutaecarpa [12] has been used in traditional Chinese medicine for hundreds of years. In addition to treating migraines, Evodia rutaecarpa is widely used in the treatment and prevention of chronic diseases such as diabetes, cardiovascular disease, and cancer [13]. The main active components of Evodia rutaecarpine are evodiamine (Evo) and rutaecarpine, which have similar structures and functions [14, 15].

Recent studies have revealed that Evo has a variety of pharmacological effects, including anti-inflammatory [16], anticancer [17, 18], antimicrobial [19], neuroprotective [20], cardioprotective [21], and therapeutic protective [22, 23] activities. Rutaecarpine has antiplatelet activation and antithrombotic effects [15, 24, 25]. Recent research results suggest that rutaecarpine promotes PI3K/Akt/GSK3 *β* signal-axis-inhibited collagen-induced platelet activation and inhibits the formation of mouse microvascular thrombosis [26]. Although the antithrombotic and antiplatelet effects of Evo have not been thoroughly investigated.

The current investigation into the antithrombotic and antiplatelet properties of Evo investigated the effects of Evo on platelet aggregation and release induced by various activators, as well as on bleeding and thrombosis in mice. Our findings showed that Evo has anticollagen-induced platelet activation ability as well as the ability to inhibit the collagen-mediated SFKs/Syk/Akt/PLC*γ*2 signal pathway. In vivo studies show that Evo has no effect on bleeding in mice, but it can significantly inhibit mesenteric thrombosis caused by ferric chloride. Our research indicates that Evo possesses antithrombotic and antiplatelet properties. Evo is anticipated to be effective as an antithrombotic and antiplatelet drug for the treatment and prevention of thrombotic diseases.

## 2. Results

### 2.1. Evodiamine Selectively Inhibits Collagen-Induced Platelet Aggregation

After the arterial endothelial injury, collagen and VWF under the endothelium are exposed to activated platelets in the blood circulation, where they induce platelet adhesion, aggregation, and activation and initiate platelet clot formation [4]. The effects of Evo on collagen-induced platelet aggregation were investigated. As shown in Figures 1(a) and 1(g), Evo inhibited collagen-induced platelet aggregation, as less than 10% platelet aggregation was observed at 50 *μ*M concentration, and the degree of inhibition was dose-dependent. After platelet aggregation, thrombin, ADP, and TXA2 were secreted and further activated platelets, thereby accelerating platelet aggregation and thrombosis in the blood circulation [27]. U46619, an activator of thrombin, ADP, and the TXA2 pathway, can also be used as platelet activators that act via various membrane receptors. The effects of Evo on the platelet aggregation induced by these activators were also investigated. Figures 1(b)–1(f) demonstrate that Evo had no discernible effect on the platelet aggregation induced by thrombin, ADP, or TXA2. As a result, we concluded that Evo primarily inhibits collagen-induced platelet aggregation.

### 2.2. Study of the Toxicity of Evo to Platelets

In recent years, it was discovered that Evo inhibits the metastasis of tumor cells, but recent studies have also revealed that it is toxic to cardiomyocytes [28]. LDH is a soluble substance that is released into the periphery when cells are damaged and can effectively reflect the toxicity of substances to cells. As a positive control, LDH was effectively released when platelets were treated with the membrane detergent Triton X-100 [29]. We investigated the effects of various Evo concentrations on platelet LDH release. The results showed that, compared with DMSO treatment, Evo below 100 *μ*M did not significantly increase platelet LDH release within 1 hour, and 250 *μ*M Evo only slightly increased the release of platelet LDH (Figure 1(h)). Accordingly, we found that under the conditions of our experiments, Evo did not cause any observable toxicity to platelets.

### 2.3. Evodiamine Inhibits Platelet Release of *α*-Granules and Dense Granules

After activation, platelets release dense granules and *α*-granules. The release of particular dense granules, such as ATP/ADP, and the expression of CD63 or LAMP-2 are regarded as specific markers of platelet activation [30]. P-selectin on the surface of platelets was detected utilizing flow cytometry. The expression of ATP and the release of ATP were detected by chemiluminescence (*α*-granules). As shown in Figure 2, collagen, ADP, U46619, and thrombin stimulated the release of granules by platelets. In comparison to DMSO treatment, Evo inhibited the release of ATP by collagen-stimulated platelets with less than 10% ATP released at 50 *μ*M (Figures 2(a) and 2(b)) and the expression of platelet P-selectin by collagen-stimulated platelets (Figures 2(d) and 2(e)). Furthermore, Evo had no significant effect on the expression of platelet P-selectin or release of ATP by ADP-, U46619-, and thrombin-stimulated platelets (Figures 2(c) and 2(f)). Thus, Evo can significantly inhibit the release of platelet granules induced by collagen.

### 2.4. Evodiamine Inhibits Collagen-Induced SFKs/Syk/PLC*γ*2 Signal Transduction

The preceding findings indicate that Evo significantly inhibits the aggregation and release of platelets induced by collagen. The major pathway for collagen-mediated platelet activation is ITAM signal transduction in platelets [31]. Therefore, we investigated the effect of Evo on platelet ITAM signaling molecules induced by Src, Syk, Akt, and PLC2 phosphorylation. The expression of immunoreceptor tyrosine-based activation motif (ITAM) signal pathway molecules in Evo-treated platelets did not differ significantly from the DMSO-treated group, as depicted in Figures 3(a) and 3(b). After collagen stimulation of platelets, the phosphorylation of ITAM signal molecules was significantly increased compared to the DMSO control group, and Evo significantly inhibited the phosphorylation of Src, Syk, Akt, and PLC following collagen activation (Figures 3(a) and 3(b)). Additionally, Evo affected the collagen-activated platelet Akt downstream signal molecule GSK-3*β*. Evo inhibited the GSK-3*β* phosphorylation process (Figure 3(c)). MAPKs consisted of the extracellular signal-regulated kinase (ERK)1/2, JNK1/2, and p38, which are also signaling molecules mediated by collagen GPVI. As depicted in Figures 3(d) and 3(e), collagen-stimulated platelet aggregation results in significant activation of JNK1/2 and p38, whereas Evo had no noticeable effect on the phosphorylation of the aforementioned MAPKs. The results demonstrated that Evo inhibits collagen-induced activation of the SFKs/Syk/Akt/PLC*γ*2 signal pathway in platelets.

### 2.5. Evodiamine Inhibits Mesenteric Artery Thrombosis In Vivo

Experiments conducted in vitro revealed that Evo significantly inhibited collagen-induced platelet activation but had no significant effect on thrombin-, U46619-, or ADP-induced platelet activation. The effect of Evo on coagulation function in mice was then investigated. According to Figure 4(c), Evo had no significant prolongation effect on tail hemorrhaging in mice, implying that Evo has little effect on the coagulation system under the conditions of this experiment. Subendothelial collagen and other matrix components are exposed to the blood during vascular endothelial injury. Platelet adhesion and aggregation on these matrix components are a critical step in the initiation of acute arterial thrombosis [32]. Therefore, we used ferric chloride to induce acute mesenteric endothelial injury and thrombosis in mice and then examined the effect of Evo on thrombosis in vivo. According to Figures 4(a) and 4(b), Evo significantly prolonged mesenteric artery embolization and inhibited thrombus volume increase when compared to DMSO treatment. As a result, Evo not only had a negligible impact on the function of coagulation but also effectively inhibited thrombosis in vivo.

## 3. Material and Methods

### 3.1. Chemicals and Reagents

Biological materials and reagents were acquired as follows: antibodies against Src, phospho-Src (Tyr416), phospho-Akt (Thr308), Akt, Syk, phospho-Syk (Tyr525/526), GSK-3*β*, phospho-GSK-3*β* (Ser9), PLC*γ*2, phospho-JNK (Thr183/Tyr185), JNK, p38 MAPK, and phospho-p38 MAPK (Thr180/Tyr182) were purchased from Cell Signaling Technology Inc. (Danvers, MA, USA). Phospho-PLC*γ*2 (Tyr 759) was acquired from GeneTex (Irvine, California, US). Peroxidase-labeled antibodies to rabbit IgG were obtained from SeraCare (Milford, MA, USA); *β*-actin was acquired from GeneTex (Irvine, CA, USA); PageRuler Prestained Protein Ladder from ThermoFisher Scientific (Shanghai, China); 5× SDS-PAGE Sample Loading Buffer and BCA Protein Assay Kit from Biosharp (Hefei, Anhui, China); polyvinylidene difluoride (PVDF) membranes from MilliporeSigma (Burlington, MA, USA); and electrochemiluminescence (ECL) western blotting detection reagent, SDS-PAGE Gel Preparation Kit, Primary Antibody Dilution Buffer, Secondary Antibody Dilution Buffer, and Western Blocking Buffer from Beyotime Biotechnology (Shanghai, China).

### 3.2. Study Protocol

The study protocol was approved by the Ethics Committee of Kunming Medical University and the First Affiliated Hospital of Kunming Medical University (Kunming, China; Approval nos. 2021-737 and 2020-L-17).

### 3.3. Platelet Aggregation and ATP Release Assay

Human apheresis platelets were obtained from healthy individuals who had not taken medication within the previous 14 days. Blood was extracted from the elbow vein of all volunteers and anticoagulated with 3.8% sodium citrate in anticoagulant tube [33, 34]. The dilution ratio of anticoagulant to venous blood was 1 : 9. Platelet-rich plasma (PRP) was separated by centrifuging acquired venous blood at 100 × g for 10 minutes at room temperature. Platelet precipitation was obtained by adding PGE1 at a final concentration of 50 ng/ml and 5 mm EDTA to the PRP, which was then centrifuged at 2000 × g for 2 minutes. Platelets were precipitated by employing Tyrode's buffer (20 mm 4-(2-hydroxytyl)-1-piperazineethanesulfonic acid [HEPES], pH 7.4, 128 mM NaCl, 12 mm NaHCO_3_, 5 mm D-glucose, 0.4 mm NaH_2_PO_4_, 2.8 mM KCl, 0.25% bovine serum albumin [BSA]) with 50 ng/ml PGE1 and 5 mm EDTA. Platelets were resuspended in Tyrode's buffer for 2 minutes to obtain washed platelets, and the platelet count was adjusted to 150 − 200 × 10^9^ platelets/L with Tyrode's buffer. The platelet aggregation experiment was carried out using a Lumi aggregometer (Chrono Log Corp.), and 1 mM calcium chloride was added to the platelet suspension before the aggregation experiment. For Fc *γ* RIIa-mediated platelet aggregation, the washed platelets were first mixed with IV.3 (1.25 *μ*g/mL) while stirring at 1200 rpm per min for 1 minute, and then, 20 *μ*g/mL of GAM IgG F(ab′) 2 antibody was added. Before the aggregation experiment, luciferin and D-luciferase were added to the platelet suspension to initiate the bioluminescence reaction [33]. The platelet activator was added after 2 minutes of incubation. The release of platelet ATP was observed using a Lumi aggregometer (Chrono Log Corp.).

### 3.4. Platelet Cytotoxicity Assay

The LDH cytotoxicity assay kit (Beyotime Biotechnology) was used to detect the platelet toxicity of Evo. First, wash platelets (200 × 10^9^/L) were incubated with various concentrations of Evo, DMSO, or 0.1% Triton X-100 (cell lysis buffer) at 37°C for 30 minutes, followed by centrifugation at 2000 × g for 10 minutes to obtain the supernatant. The supernatant was treated according to the instructions, and the absorbance value was measured at 490 nm using a Multiskan FC (ThermoFisher Scientific Inc., Waltham, MA, USA) spectrophotometer.

### 3.5. Flow Cytometry

Washed platelets (50 × 10^7^/L) were incubated with various concentrations of Evo, DMSO, or PGE1 for 10 minutes at 37°C. Platelets were washed after incubation, 1 mM calcium chloride and platelet agonist were added, and 10 mm EDTA was added 30 minutes later to stop the reaction. Platelets were incubated with phycoerythrin- (PE-) conjugated anti-cd62p (P-selectin) monoclonal antibody for 30 minutes, and then, the fluorescent-labeled platelets were detected by flow cytometry in a Facscanto II flow cytometer (BD Biosciences, San Diego, CA, USA).

### 3.6. Western Blotting

Platelets were resuspended in Tyrode's buffer B without 0.25% BSA and incubated at 37°C for 5 minutes with DMSO (vehicle group) or Evo. Processed platelets were stimulated with Evo before 2 × Triton X-100 cell lysis buffer (PBS, pH 7.4, comprising 10 mM EDTA, 145 mM NaCl, 2 × 0.5% sodium dodecyl sulfate [SDS], 2 × 1% deoxycholate, 2 × 1% vol/vol Triton X-100, 2 × phosphatase, and proteinase inhibitors cocktails) was added for 60 seconds. The treated platelets were centrifuged at 12000 × g for 10 minutes, and the supernatant was retained. The concentration of the protein was measured by employing a BCA protein assay reagent after heating at 100°C for 10 minutes. 5× SDS-PAGE sample loading buffer was added after protein quantification. The platelet lysate was loaded and separated using a 10% (wt/vol) sodium dodecyl sulfate-polyacrylamide gel electrophoresis (SDS-PAGE) gel. The separated peptides were subsequently transferred onto PVDF membranes. Tris-buffered saline with Tween (TBST) containing 20 mM Tris, 137 mM NaCl, and 0.1% Tween-20 was used to rinse the membranes three times. After blocking the PVDF membranes with blocking buffer at 4°C for 1 hour and washing with TBST once, the membranes were incubated during the night hours at 4°C with primary antibodies diluted in primary antibody dilution buffer. Src, Syk, Akt, PLC*γ*2, GSK-3*β*phospho-Src, phospho-Syk, phospho-Akt, phosphor-PLC*γ*2, phosphor-GSK-3*β*, and *β*-actin were detected by implementing particular antibodies at a dilution ratio of 1 : 1000. Following rinsing with TBST three times, the membranes were incubated for 3 hours at 4°C with a peroxidase-labeled antibody to rabbit IgG, which was employed as a secondary antibody at a dilution ratio of 1 : 5000. The target protein bands were visualized using ECL after antibody incubation and three washes with TBST. The intensity of the target bands was assessed by ImageJ software.

### 3.7. Mouse Tail Hemorrhage Experiment

C57/b6l mice aged 6-8 weeks were anesthetized with sevoflurane. The coagulation time was then measured by placing a 5 mm sample of the mice's tails into normal saline at 37°C. Blood coagulation was assumed to have occurred when there was no blood flow for 60 s.

### 3.8. Ferric Chloride-Induced Mesenteric Thrombosis in Mice

C57/b6l mice aged 6-8 weeks were anesthetized by an intraperitoneal injection of pentobarbital (45 mg/kg). After the mice were fixed in position, the neck hair was cut off, the neck skin was cut open, the jugular vein was found and catheterized, and rhodamine (5 mg/kg) was injected. The abdominal cavity was opened to expose the mesenteric vessels, and mesenteric arterioles with a diameter of about 60-80 *μ*M were selected under the microscope. Filter paper (approx. 5 mm long and 2 mm wide) soaked in 7.5% FeCl_3_ solution was placed on blood vessels for 2 minutes to induce vascular injury and thrombosis. Evo (10 mg/kg) or DMSO was injected into the jugular vein 30 minutes before thrombosis induction. Images were captured every 5 minutes using an MSHOT MD50 camera (Micro Shot Technology Ltd., Guangzhou, China) and an Olympus ix73 microscope (Olympus Corp., Shinjuku, Japan) during thrombosis. More than 90% of the blood vessels were considered completely occluded, and the longest observation time was 80 minutes.

### 3.9. Statistical Analysis

All experimental results were analyzed with GraphPad 5.0 Prism software and presented as the mean ± standard error of the mean (SEM). A two-tailed unpaired comparison *t*-test was utilized for comparing differences between two experimental groups. To compare more than two groups, we used a one-way analysis of covariance (ANOVA). The significance level was considered at *P* < 0.05.

## 4. Discussion

Evodia rutaecarpa has multiple pharmacological effects and is widely used in the treatment and prevention of chronic diseases such as migraines, diabetes, cardiovascular disease, and cancer [35]. Although the antithrombotic and antiplatelet effects of Evo remain unclear. We discovered that Evo significantly inhibited the aggregation of collagen-activated platelets, but had no significant effect on platelet activation induced by other activators, including thrombin, ADP, and U46619. Furthermore, Evo had no significant toxic effects on platelets at the dose described in Figure 1. In addition, the *α*-granule- and dense-granule-release experiments confirmed the selective inhibitory impact of Evo on collagen-induced platelet activation (Figure 2). According to the signal pathway analysis, Evo inhibited collagen-induced platelet ITAM-signal transduction (Figure 3). In vivo experiments also confirmed that our experimental dose of Evo did not significantly affect the bleeding time of mice, but it significantly prolonged the mesenteric thrombosis induced by ferric chloride (Figure 4). The results of the current study show that Evo can be used as an effective antiplatelet medication to inhibit platelet activation and thrombosis. Atherosclerotic plaque rupture or vascular endothelial cell injury is the main pathological change leading to acute thrombosis [36]. Following vascular wall injury caused by shear stress in the artery, collagen and VWF are exposed to the bloodstream and interact with platelets. The blood platelet membrane protein GPib-v-ix mediates acute adhesion of platelets to the injury surface [6]. The interaction between platelet membrane proteins and collagen performs an essential task in the formation of platelet clots on the damaged surface of the endothelium in the early stages of thrombosis [37]. The results showed that Evo significantly inhibited the aggregation and release of collagen-induced platelets, but had no effect on the aggregation and release of ADP-, U46619-, and thrombin-induced platelets. As a result, we hypothesized that Evo exerts its inhibitory antiplatelet-aggregation function primarily through collagen-platelet interactions. According to several investigations, it has been found that the adhesion between platelets and collagen is dependent on the collagen receptors GPVI, *α*2*β*1, and GPIb-IX-V and that the activation process after platelet adhesion is mostly mediated through GPVI—an important collagen receptor of platelets [4, 37]. In the physiological state, GPVI and FCR*γ* form a heterodimer, and GPVI uses the ITAM base sequence of FcR*γ* to transduce intracellular activation signals [38].

We also discovered that Evo had a negligible effect on collagen receptor-mediated platelet aggregation induced by the GPVI-specific activator convulxin (results not shown). Although GPVI, as the primary receptor of collagen, mediates platelet activation and adhesion, platelet activation is mediated by a network of membrane receptors that interact with collagen in a vertically and horizontally intertwined activation network [37–39]. Therefore, Evo may act on receptors other than GPVI receptors, such as the *α*2*β*1 receptor, which mainly mediates the early activation of platelets. In combination with secondary activation receptors on platelets, *α*2*β*1 can further activate the main platelet collagen receptor GPVI. A monoclonal antibody that inhibited its effect significantly reduced the aggregation of collagen-induced platelets [40]. Consequently, based on current experimental findings, Evo may also influence *α*2*β*1-mediated platelet activation function; however, the specific mechanism remains to be determined.

The tyrosine of the intracellular segment of FcR*γ*'s ITAM sequence is phosphorylated when GPVI is activated by its ligand. This phosphorylated site can recruit and bind to the SH2 domain of Syk, which can then be activated by itself or SFKs [41, 42]. The activation of Syk triggers the phosphorylation of lat, a downstream signal-transduction member. After lat is activated, it can phosphorylate a variety of signal molecules, such as PI3K, SLP-76, Grb2, and SHC, which leads to PLC*γ*2 activation [43–45]. The activation of PI3K combined with lat acts on PIP2 and generates PIP3. PIP3 is enriched by Btk and Tec and activated by phosphorylated PLC*γ*2. Activated PLC*γ*2 decomposes phospholipids to produce the second messengers IP3 and DAG, which cause the increase of calcium from platelets and the activation of PKC [43, 45].

The analysis of signal transduction results revealed that Evo significantly inhibited the collagen-mediated platelet ITAM signal pathway molecules Src, Syk, and PLC *γ*2 (Figures 3(a) and 3(b)). Based on the findings presented above, we have concluded that Evo exerts a significant inhibitory effect on collagen-mediated platelet activation and that its mechanism is primarily associated with the SFKs/Syk/PLC *γ*2 signal pathway.

The serine/threonine kinase Akt is an important effector molecule of PI3K, and PI3K/Akt also performs an essential regulatory task in GPVI-mediated signal transduction. Akt-knockout mice show defective platelet activation [46], and the Akt regulator GSK3 *β* is also regarded as necessary for platelet activation [47]. Previously, it was discovered that the arterial thrombotic instability of platelet-specific PI3K-*β*-deficient mice was superior to that of wild-type mice under conditions of high shear stress. This may be due to the inhibition of Akt and GSK3 functions during thrombotic enlargement [47]. According to the findings of this study, the degree of phosphorylation of Akt and GSK3 GSK3*β*, which are activators of the PI3K signaling pathway, is very low in platelets when they are in their resting state (Figures 3(a)–3(c)). Following stimulation with collagen, there was a notable increase in the degree to which Akt and GSK3*β* were phosphorylated, and Evo was found to have a significant inhibitory effect on their phosphorylation (Figures 3(a)–3(c)).

The results of previous studies suggest that PI3K/Akt and MAPKs activate each other within platelets. MAPKs are comprised of a group of serine/threonine kinases that are capable of translating extracellular stimuli into cellular responses [48]. MAPK family members include ERK1/2, p38 *α*, *β*, *γ*, and *δ*, JNK1/2/3, and big MAPK (ERK5). Several investigations employing MAPK-specific inhibitors or MAPK knockout in mice demonstrated that ERK1/2, JNK1/2, and p38 MAPK are present in platelet activation and thrombosis [48–50]. We found that Evo demonstrated no significant inhibitory impact on the phosphorylation of MAPK family molecules p38 and JNK1/2 (Figures 3(d) and 3(e)). Recent research results suggest that rutaecarpine, another extract of Evo, works through PI3K/Akt/GSK3*β* and the MAPK signal axis to inhibit collagen-induced platelet activation. The findings of this study indicate that Evo inhibits the collagen-induced SFKs/Syk/Akt/PLC*γ*2 inhibition of the platelet activation signal pathway. In conjunction with other research, the results of this investigation have led us to hypothesize that the effect of Evodia rutaecarpa extract on collagen-induced platelet activation is achieved through a combination of different signal transduction pathways.

One of the most important steps in the development of acute arterial thrombosis is the adhesion and aggregation of platelets, which takes place when platelets are subjected to a strong shearing force [27]. The mouse mesenteric thrombosis induced by ferric chloride mimics the pathophysiology of human atherosclerotic plaque rupture and thrombosis and is a widely used animal experimental model for evaluating platelet function and observing arterial thrombosis [51, 52]. Furthermore, blocking the collagen receptor GPVI with a monoclonal antibody can significantly reduce the mesenteric thrombosis induced by ferric chloride in mice [53, 54]. This model was chosen to examine the effect of Evo on thrombosis in vivo based on the in vitro experimental findings of the current work (Figures 4(a) and 4(b)). It was discovered that iron chloride significantly increased the bleeding time of Evo-treated mice. This experiment, however, had limitations. We did not observe thrombosis induction for a long time, and recent studies revealed that the mechanism of thrombosis in this mouse model is closely related to many factors, including ROS injury of endothelial cells, erythrocyte adhesion, and the role of plasma proteins [55, 56]. To further investigate the mechanism of Evo's effect on thrombosis, fluorescent staining and microscopy are required to observe the interactions between cells during the thrombosis process.

Although this study suggests that the effects of Evo on platelets are linked to collagen, the platelet membrane proteins that interact with Evo were not identified. Evo inhibits collagen-induced platelet activation but has a negligible effect on GPVI-mediated platelet aggregation. These experimental results led us to suspect that Evo acts through other collagen receptors such as *α*2*β*1 and GP Ib-V-IX, which may interact to play an antiplatelet role. To further investigate the effects of Evo on platelet *α*2*β*1 and GPIb-V-IX function, it is necessary to improve this investigation of the adhesion between platelets and collagen subjected to static and high shear forces. Furthermore, Evo exhibits anti-inflammatory and antioxidant properties [57]. The effects of Evo on platelet activation, apoptosis, autophagy, and other functions under oxidative stress are also worthy of further investigation. In vitro studies demonstrated that Evo selectively inhibits collagen-induced human platelet activation. According to the in vivo findings, Evo significantly inhibited the thrombosis induced by ferric chloride while not significantly prolonging bleeding time. However, it is necessary to pay attention to the complex pathological processes of thrombosis, as well as the inhibitory effects of Evo on endothelial cells and neutrophils. It is still worthwhile to investigate whether Evo has significant inhibitory effects in several different types of pathological thrombosis, such as venous embolism and tumor embolism, and so on. As a Chinese patent medicine with multiple activities, Evo appears to have effects on platelets and thrombosis, and the current work has provided a novel experimental foundation for the investigation of the pharmacological mechanism of Evo and the development of antiplatelet and antithrombotic drugs.

In conclusion, the effects of Evo on antiplatelet activation and thrombosis were investigated in this study, and it was demonstrated that Evo effectively inhibited collagen-induced platelet activation but had no effect on platelet aggregation caused by activators such as thrombin, ADP, and U46619. In addition, the effect of Evo on the release of platelet granules was studied, and the results demonstrated that Evo can effectively inhibit the release of platelet granules induced by collagen. It can also significantly inhibit the collagen-mediated SFKs/Syk/Akt/PLC*γ*2 signal pathway. In vivo studies on the mesenteric artery, thrombosis revealed that the Evo has no effect on bleeding in mice, but it can significantly inhibit ferric chloride-induced mesenteric thrombosis. This study found that Evo has antithrombotic and antiplatelet properties and that it can be used effectively as an antithrombotic and antiplatelet drug for the treatment and prevention of thrombotic diseases.

## Figures and Tables

**Figure 1:** Evodiamine toxicity and effect on the aggregation of platelets caused through diverse activators.

**Figure 2:** Influence of evodiamine on collagen-induced platelet dense granule and *α*-granule release.

**Figure 3:** Influence of Evo on collagen-induced platelet ITAM-activation signal pathway.

**Figure 4:** Influence of evodiamine on thrombosis and hemostatic function induced by ferric chloride.

## Data Availability

Data will be provided upon request to the authors.
